This article has been retracted.

# Analysis of Etiology and Risk Factors of Catheter-Associated Urinary Tract Infection in Critically Ill Patients and Research on Corresponding Prevention and Nursing Measures

**DOI:** 10.1155/2021/8436344

**Published:** 2021-12-20

**Authors:** Du Juanjuan, Zhao TianTian, Dong Yue, Wang Lili, Xu Ping, Hongyun Xu

**Affiliations:** ^1^China Lianyungang City First People's Hospital, Lianyungang Hospital Affiliated to Xuzhou Medical University, Lianyungang, Jiangsu Province 222000, China; ^2^Two Departments of Critical Care Medicine, Anhui Wanbei Coal-Electricity Group General Hospital, Suzhou, 234000 Anhui, China

## Abstract

Catheter-associated urinary tract infection (CAUTI) is the most common complication in patients with indwelling catheterization. The incidence of CAUTI in my country is still at a relatively high level compared with foreign countries, especially for the ICU, which has a high usage rate of urinary catheters, to focus on prevention and control. This article focuses on studying the risk factors of CAUTI in critically ill patients and discusses targeted preventive care measures. This article investigates and examines the clinical data of CAUTI in critically ill patients. After statistical analysis, the risk factors that affect CAUTI are summarized, so as to derive the cause of CAUTI in order to strengthen clinical care and to further study the prevention, control, and nursing of CAUTI to provide reference. Clinical data shows that the CAUTI infection rate of patients with catheter indwelling ≥7 days is greater than that of patients with catheter indwelling days less than 7 days. The CAUTI infection rate of the patients who change the urine collection bag every day or ≥7 days is greater than that of the patients who change the urine collection bag within 2 to 4 days.

## 1. Introduction

CAUTI refers to the urinary tract infection that occurs in patients after the catheter is indwelled or within 48 hours after the catheter is removed [1, 2]. Residential catheterization is a common method in clinical practice. This requires not only testing this condition, but is a major measure for certain diseases. The most common and important complication is the CAUTI. It is also one of the most common infections in the world [3, 4]. CAUTI not only affects the success rate of patient treatment, but is also the main reason for the prolonged hospitalization time and the substantial increase in hospitalization costs [5, 6]. At the same time, the occurrence of CAUTI seriously affects hospital's reputation, reputation, brand, and sustainable development. Occupational exposure increases the risk of infection among medical staff [7, 8]. Therefore, the study of CAUTI risk factors for critically ill patients is of great significance.

Regarding the research of CAUTI, many scholars at home and abroad have conducted in-depth discussions. For example, Roy et al. found through research that if the recommended preventive measures are taken, the occurrence of CAUTI can be reduced [9]; Muramatsu et al. noted that clinics should focus on the training of caregivers and standardize the operation of catheter care to reduce the incidence of CAUTI caused by iatrogenic factors [10].

This article focuses on studying the risk factors of CAUTI in critically ill patients and discusses targeted preventive care measures. This article investigates and examines the clinical data of CAUTI in critically ill patients. After statistical analysis, the risk factors that affect CAUTI are summarized, so as to derive the cause of CAUTI in order to strengthen clinical care and to further study the prevention, control, and nursing of CAUTI to provide reference.

## 2. Risk Factors for CAUTI in Critically Ill Patients

### 2.1. Risk Factors for Catheter-Related Urinary Tract Infection in Critically Ill Patients

#### 2.1.1. The Longer the Catheter Is Indwelled, the Higher the CAUTI Infection Rate

With the extension of permanent catheters in ICU patients, the incidence of CAUTI also increases. This is because the permanent urinary catheter destroys the normal environment of the urethra, and the immune system weakens the phagocytosis of neutrophils, which affects the physiological role of the bladder on bacteria, making it easier for bacteria to enter the bladder and ureter, and the development of organs in the system and reproduction can cause infection [11, 12]. At the same time, bacterial biofilms formed by bacteria on the urethral surface increase bacterial resistance to antimicrobial agents and host immune function, leading to fever, urethral stimulation, bladder inflammation, and even, urethral-associated infections. Thus, urine is internal, and although the catheter can prevent and treat various diseases, it is more likely to cause CAUTI.

In other words, for patients with long-term indwelling catheters, frequent replacement of catheters may be more likely to cause urinary tract infections, so the most appropriate replacement method is generally to replace the patient when the patient has an infection or the catheter is blocked.

#### 2.1.2. The Infection Rate of CAUTI in the Elderly Is Higher

After processing the survey data, the impact of patient age distribution on CAUTI is shown in Table 1. The incidence of CAUTI in patients younger than 30 years old with indwelling catheters is 10%, and the incidence of CAUTI in patients aged 30, 40, and 50 years old is about 10%. They are 10%, 22.22%, 25%, and 25%, respectively (*x*^2^ = 7.21, *P* < 0.05).

It can be seen from Figure 1 that the older the age, the greater the incidence of CAUTI, so the incidence of CAUTI in the elderly is higher.

With age, the body's physiological defense function gradually decreases, and the functions of important organs in the elderly ≥60 years old gradually deteriorate, making them susceptible to CAUTI. At the same time, most elderly people are accompanied by serious chronic diseases. Once invasive operations such as catheterization are performed, the immune defense function of the whole body will be damaged, the resistance will be greatly reduced, and the susceptibility to diseases will be greatly increased.

CAUTI can severely affect the quality of life of elderly patients and increase the time of hospital stay and medical expenses. Therefore, the principle of aseptic surgery should be strictly adopted in the treatment and care of elderly patients to reduce unnecessary invasive surgery. Multiple methods can be used to improve the immune function in elderly patients and reduce the morbidity.

#### 2.1.3. Analysis of Changing Time of Urine Collection Bag

The comparison of CAUTI infection rates with different urine collection bag replacement time is shown in Table 2: when the urine collection bag replacement time is 1 day, the CAUTI incidence rate is 25.93%; when the urine collection bag replacement time is 2 to 4 days, the CAUTI infection rate is 13.33%. (*x*^2^ = 5.24, *P* < 0.05).

It can be concluded from Figure 2 that patient's urine collection bag replacement time is best 2 to 4 days, and patient's daily urine collection bag replacement or replacement urine bag time is ≥7 days, which significantly increases the incidence of CAUTI in patients with indwelling catheters.

Changing the urine collection bag every day will artificially destroy the closed drainage system and easily contaminate the connection between the urine collection bag and the urinary catheter, resulting in a significant increase in the infection rate of CAUIT. The urine collection bag replacement time is ≥7 days. The urine is prone to turbidity and crystallinity, which increases the probability of urethral obstruction. It is easy to cause bacterial viruses and other pathogenic microorganisms to multiply, which directly leads to an increase in the CAUIT infection rate. Therefore, the best time to replace the urine collection bag is 2 to 4 days.

#### 2.1.4. Replacement Time of Urinary Catheter

Patient's catheter replacement time should best be replaced every 2 weeks. By extending the mounting time of the catheter, a bacterial biofilm will be formed on the surface of the catheter to facilitate the adhesion and reproduction of bacteria and viruses. Bacterial biofilms can protect bacteria and viruses from host immune responses and eliminate bacteria. Therefore, it would be difficult to remove the source of infection without pulling out or replacing the catheter.

### 2.2. CAUTI Prevention and Care

#### 2.2.1. Management and Supervision

Medical institutions need to set up full-time management personnel to formulate and update the detailed rules for the application of cluster management to prevent CAUTI in critically ill patients and regularly conduct publicity and education, skill training, implementation inspections, and effect evaluations for medical staff. At the same time, the necessary medical conditions are provided for cluster management. At least each ward should have a handwashing basin, and each bedside should be equipped with disinfectant.

#### 2.2.2. Hand Hygiene Throughout

The implantation of the catheter should be performed by a qualified physician. The hands should be cleaned with soap or hand sanitizer before the operation, and sterile gloves should be worn during the operation; hands should be cleaned before and after the catheter is used and before and after changing the dressing of the puncture site, if possible. It is best to wear clean or sterile gloves; when the catheter is pulled out, it is recommended to wear sterile gloves to avoid infection caused by bacteria passing through the puncture point due to contact.

#### 2.2.3. Requirements for the Intubation Process

Surgeons should wear masks, hats, sterile gloves, sterile surgical suits, and use sterile masks covering patient's whole body to reduce the number of observers. The optimal catheter location and type of catheter were selected based on patient's own condition. For patients with high risk of infection, a catheter coated with heparin or antibiotics can be used. It is recommended to cover the puncture site with a transparent dressing or sterile gauze after surgery. Transparent dressing is more convenient to observe the puncture point than sterile gauze and contributes to the timely detection of infection signs.

#### 2.2.4. Use and Care of Catheter

The choice of catheter type and material depends on the size of patient's urethra and clinical judgment. Generally, hydrophilic materials are selected. Urinary catheters should be thoroughly disinfected before and after use to avoid multiple uses of one tube. After dialysis, the residual urine in the catheter should be flushed with normal saline. Patients with high risk of infection or suspected CAUTI patients should be given antibiotics and sealed with sterile gauze. Evaluate whether the catheter continues to be retained every day, and pull out the catheter that is no longer in use in time. At the same time, patient's body temperature should be monitored every day to facilitate timely detection and treatment of CAUTI.

### 2.3. Capillary Electrophoresis to Detect Urinary Tract Bacteria

Capillary electrophoresis, as a new high-efficiency separation technology, is developed on the basis of traditional electrophoresis. The basic theory lies in the transfer of solutes in the capillary zone electrophoresis process. Electrophoresis is the directional movement of charged particles under the action of an electric field. The electrophoresis rate (*v*/*E*) under a unit electric field is called mobility or electric mobility (*μ*_*ep*_), and the mobility measured in an infinitely diluted solution is called absolute mobility *μ*^0^_*ep*_. Under the action of the electric field, the electric field force received by the dotted particle *F*_*e*_ is equal to the product of its static charge *q* and the electric field strength *E*, namely.

(1) $$\begin{array}{c} F_{\text{e}}=q\cdot E, \end{array}$$

(2) $$\begin{array}{c} E=\frac{\bar{U}}{L}, \end{array}$$

where $\bar{U}$ is the DC voltage applied across the capillary and *L* is the length of the capillary.

## 3. Experimental Study on Risk Factors of CAUTI in Critically Ill Patients

### 3.1. Research Objects

Patients who were selected to be admitted to the intensive care unit of Hospital H on October 6, 2019, include patients who were discharged, transferred, or died on the same day and do not include patients who were admitted to the hospital on the day of the investigation. Patients were collected through a combination of bedside surveys and hospital events. Patients who used permanent catheters after urinary tract infections and those who had used permanent catheters at the time of admission were excluded. In the end, a total of 70 patients participated in the investigation of this study.

### 3.2. Research Methods

#### 3.2.1. Questionnaire

The survey content consists of four parts:

1. General information of the patient: according to the gender of the patient, they are divided into male and female groups, and the infection rates of CAUTI are calculated, respectively. According to the age of patients, <30, 30~, 40~, 50~, and ≥60 five levels analyze the relationship between age and CAUTI infection rate

The number of days hospitalized by case inquiry is the time of stay from the date of stay to the date of investigation. The mean length of hospitalization between the two groups was calculated based on whether they had CAUTI, to classify patients into infected and uninfected groups. Previous medical history mainly discussed whether the relationship between patients have diabetes and benign prostate hyperplasia and the CAUTI infection rate.

(2) Patient's urinary tract infection information: according to patient's state of consciousness, the CAUTI infection rate was divided into four levels: lethargy, confusion, lethargy, and coma for comparative analysis

According to patient's urine collection bag replacement time (days), it is stratified into four levels: 1, 2~4, 4-6, and ≥7; according to the urinary catheter replacement time (weeks), the stratification is 1, 2, and ≥4 three levels.

### 3.3. Quality Control

Before collecting data, conduct intensive training for investigators. The investigators included 4 postgraduates from the nosocomial infection research group and 3 postgraduate nurses in neurosurgery of the hospital. The training content includes investigation methods, data collection, knowledge about CAUTI infection, treatment, and nursing knowledge and skills.

### 3.4. Methods of Data Collection

#### 3.4.1. General Patient Data Collection Method

The investigator himself screened patients with indwelling catheters, explained the purpose, methods, and rights of the study to eligible patients, and obtained their patients' informed consent before they were included in the study. In this study, general patient information was collected by consulting medical records and bedside inquiries.

#### 3.4.2. Collection Method of CAUTI Infection Rate Data

The investigator kept a urine specimen on the day the catheter was removed. The method is before removing the urinary catheter, disinfect the sampling point with a cotton swab soaked in the urinary tube (if there is no sampling point in the catheter, the “Y” of the disinfected urinary catheter should be bifurcated downwards, and the nonsaccharide filling port upwards 3 cm away), draw 510 ml of urine from the catheter with a sterile syringe, and inject it into the sterile specimen cup. After collecting the urine sample, immediately send it to the laboratory for culture test. For patients with repeated catheterization, the catheter needs to be kept before removal each time.

#### 3.4.3. Analysis Methods of High-Risk Factors for Catheter-Related Infections

Before data entry of the questionnaire, the data of all the questionnaires shall be initially screened, and the questionnaires with serious missing data shall be excluded. The duo entered the data into the Excel database and repeatedly verified the proofreading data information.

### 3.5. Nursing Procedures Related to Urinary Catheters

#### 3.5.1. Indwelling Urinary Catheter

Most patients in the ward who require surgical treatment require indwelling urinary catheters, except for patients who have undergone intramedullary nail removal and plate removal. On the day of the operation, before being sent to the operating room, the doctor in charge issued a medical order, and the responsible nurse performed indwelling catheterization. The indwelling guide tube is then brought into the operating room by the patient. For some male patients with enlarged prostate or elderly women with hypertrophic labia, indwelling urinary catheterization is performed by nurses in the operating room.

After completion of the operation, the patient can be transferred to ICU observation according on patient's condition or directly returned to ward's treatment. Patients transferred to ICU usually return on day 23 after surgery and after a stable condition. Following doctor's order to remove the catheter, the nurse removed the catheter 27 days after surgery. Individual patients can be hospitalized for up to 1 month.

#### 3.5.2. Catheter Care and Management

Nursing and management requirements after intubation:

1. When the patient is lying in bed, fix the urine collection bag of the urinary catheter to the bed unit with a pin to avoid discounting or bending. The height of the urine collection bag is lower than the level of the bladder to avoid contact with the ground and prevent retrograde infection
2. During the indwelling catheter, use a broken solution to clean the urethral opening, once a day in the morning and afternoon. Patients with fecal incontinence should also be disinfected after cleaning
3. According to the type of urinary catheter, short-term urinary catheters should be replaced every 7 days, and long-term urinary catheters should be replaced every 30 days
4. Change the urine collection bag every 3 days
5. Irrigation is not routinely performed, and antibiotics are not routinely used for bladder washing
6. Before removing the urinary catheter, perform clamping to train the bladder function. The method is to remove the bladder when the patient is willing to urinate after the clamping. There are also patients who are intermittently clamped according to doctor's request, open every 4 hours, and remove the catheter after 12 days of exercise

#### 3.5.3. Disposal after Infection

When nurses find suspected signs of infection such as fever, lower abdomen pain, and percussion pain in the kidney area in patients with indwelling catheterization, they should take physical measures such as cooling down and report patient's condition to the doctor in charge to assist the doctor in taking corresponding treatment and collecting urine specimens.

## 4. Data Analysis of Risk Factors for CAUTI in Critically Ill Patients

### 4.1. Impact of Catheter Replacement Time on CAUTI

The effect of catheter replacement time on CAUTI is shown in Table 3: when the catheter replacement time is 1 or 2 weeks, the incidence of CAUTI is 35.71% and 16.67%, respectively; when the catheter replacement time is 4 weeks, the incidence of CAUTI is 25%. After statistical analysis, *x*^2^ = 5.06, *P* < 0.05, the difference is statistically significant.

It can be concluded from Figure 3 that there is a significant relationship between the catheter replacement time of critically ill patients and the infection rate of CAUTI, suggesting that for patients using Foley's silicone catheters, nursing staff should replace catheters every 2 weeks tube.

### 4.2. Impact of Underlying Diseases on CAUIT

The comparison of the CAUTI infection rate of different underlying diseases is shown in Table 4. For the five major types of basic diseases in the neurosurgery department, the incidence of CAUTI between patients with different disease types is compared with the incidence of CAUTI. After *x*^2^ test, *x*^2^ = 6.91, *P* < 0.05, which is statistically significant.

From Figure 4, it can be concluded that the incidence of CAUTI in patients with cerebral hemorrhage is 36.36%, which is the first of the five basic diseases, followed by the incidence of CAUTI of craniocerebral injury at 25%, and CAUTI of intracranial tumors. The incidence rate is 20%.

## 5. Conclusion

CAUTI is one of the common complications of critically ill patients with indwelling catheter. This article focuses on studying the risk factors of CAUTI in critically ill patients, and discusses targeted preventive care measures. This article investigates and examines the clinical data of urinary CAUTI in critically ill patients. After statistical analysis, the risk factors that affect CAUTI are summarized, and the causes of CAUTI are obtained in order to strengthen clinical care, to further study the prevention, control, and nursing of CAUTI to provide reference.

## Figures and Tables

**Figure 1:** The influence of patient age distribution on CAUTI.

**Figure 2:** Influence of changing time of urine collection bag on CAUIT.

**Figure 3:** The effect of catheter replacement time on CAUIT.

**Figure 4:** The impact of underlying diseases on CAUIT.

**Table 1:** The influence of patient age distribution on CAUTI.

Patient age (years)	Number of patients	CAUTI number	Infection rate%
<30	10	1	10
30~	9	2	22.22
40~	12	3	25
50~	20	5	25
≥60	19	8	42.11
Total	70	18	25.71

**Table 2:** Influence of changing time of urine collection bag on CAUIT.

Urine bag replacement time (days)	Number of patients	CAUTI number	Infection rate%
1	27	7	25.93
2~4	30	4	13.33
4~6	7	3	42.86
≥7	6	4	66.67
Total	70	18	25.71

**Table 3:** The effect of catheter replacement time on CAUIT.

Catheter replacement time (weeks)	Number of patients	CAUTI number	Infection rate%
1	28	10	35.71%
2	30	5	16.67%
4~	12	3	25%
Total	70	18	25.71%

**Table 4:** The impact of underlying diseases on CAUIT.

Type of disease	Number of patients	CAUTI number	Infection rate%
Cerebral hemorrhage	36	11	30.55
Brain injury	12	3	25
Intracranial tumor	5	1	20
Intracranial aneurysm	8	1	12.5
Other	9	2	22.22
Total	70	18	25.71

## Data Availability

The data underlying the results presented in the study are available within the manuscript.
